The article "Computational FEM Model and Phantom Validation of Microwave Ablation for Segmental Microcalcifications in Breasts Using a Coaxial Double-Slot Antenna" was published in 2021. Journal: Biomed Res Int.

# Computational FEM Model and Phantom Validation of Microwave Ablation for Segmental Microcalcifications in Breasts Using a Coaxial Double-Slot Antenna

**DOI:** 10.1155/2021/8858822

**Published:** 2021-02-22

**Authors:** Kristian Segura Félix, Geshel D. Guerrero López, Mario F. J. Cepeda Rubio, José I. Hernández Jacquez, Francisco G. Flores García, Arturo Vera Hernández, Lorenzo Leija Salas, Eva C. Orozco Ruiz de la Peña

**Affiliations:** ^1^División de Estudios de Posgrado e Investigación, Instituto Tecnológico de la Laguna, Torreón, 27274 Coahuila, Mexico; ^2^CBTIS 196 Matamoros, 27440 Coahuila, Mexico; ^3^Sección de Bioelectrónica, Centro de Investigación y de Estudios Avanzados del Instituto Politécnico Nacional, México DF 07360, Mexico; ^4^Hospital General de Durango, Durango, 34000 Torre Materno-Infantil, Mexico

## Abstract

**Introduction:**

Cancer is the second leading cause of death worldwide. Breast cancer is the second most common cause of cancer-related mortality, accounting for 11.6% of the total number of deaths. The main treatments for this disease are surgical removal of the tumor, radiotherapy, and chemotherapy. Recently, different minimally invasive technologies have been applied (e.g., emission of electromagnetic waves, thermal and chemical means) to overcome the important side effects of these treatment modalities. The objective of this study was to develop and evaluate a predictive computational model of microwave ablation.

**Materials and Methods:**

The predictive computational model of microwave ablation was constructed by means of a dual-slot coaxial antenna. The model was compared with an experiment performed using a breast phantom, which emulates the dielectric properties of breast tissue with segmental microcalcifications. The standing wave ratio (SWR) was obtained for both methods to make a comparison and determine the feasibility of applying electromagnetic ablation to premalignant lesions in breasts. Specifically, for the analysis of segmental microcalcifications, a breast phantom with segmental microcalcifications was developed and two computational models were performed under the same conditions (except for blood perfusion, which was excluded in one of the models).

**Results:**

The SWR was obtained by triplicate experiments in the phantom, and the measurements had a difference of 0.191 between the minimum and maximum SWR values, implying a change of power reflection of 0.8%. The average of the three measurements was compared with the simulation that did not consider blood perfusion. The comparison yielded a change of 0.104, representing a 0.2% change in power reflection. *Discussion*. Both experimentation in phantom and simulations demonstrated that ablation therapy can be performed using this antenna. However, an additional optimization procedure is warranted to increase the efficiency of the antenna.

The article "Computational FEM Model and Phantom Validation of Microwave Ablation for Segmental Microcalcifications in Breasts Using a Coaxial Double-Slot Antenna" was published in 2021. Journal: Biomed Res Int.

## 1. Introduction

Cancer is the second cause of death worldwide, accounting for 18,078,957 cases and 9,555,027 deaths in 2018. The most common type is lung cancer, representing 11.6% of the total number of cases and accounting for the highest number of deaths due to cancer (18.4%). It is followed by breast cancer with 2,088,849 cases (11.6%) and 626,679 deaths (6.6%) [1]. Currently, the main treatments for cancer are the surgical removal of the tumor, chemotherapy, radiotherapy, or combinations of these modalities. However, these treatments are associated with important physical and emotional side effects [2]. Therefore, the application of different technologies (e.g., tissue ablation through the emission of electromagnetic waves, chemical or thermal means) has been investigated [3]. The one that has had the most promising results in multiple tissues such as the bone and liver is microwave ablation performed by needle applicators. Tests with different models of antennas have been carried out to optimize the treatment [4–6]. Puncture planning methods have been developed to make procedures more accurate [7], and it has been shown to be more effective and safe than other therapies. This is because it is not necessary to use a reference electrode as in the case of radiofrequency ablation; electromagnetic waves can propagate by all kinds of biological tissue. Moreover, it is possible to make arrangements of more than one antenna and presents less procedural pain [8]; and needle applicators can be produced at a low cost [9].

An important correlation has been found between the presence of premalignant lesions (segmental and linear microcalcifications) and the development of cancer since most of the patients who present this type of lesion undergo surgery, chemotherapy, or radiotherapy [10, 11]. The efficiency was studied using a double-slot antenna in the said medium, having this work as an objective to demonstrate the feasibility in the application of electromagnetic ablation by means of a computational model as well as to validate it by means of experiments in a tissue-mimicking phantom.

## 2. Materials and Methods

Microwave ablation [12–14] therapy involves the emission of high-frequency electromagnetic waves, which causes the polar molecules of water found in the tissue to rotate. This rotation generates mechanical heat, which eventually leads to cellular necrosis [14, 15]. Unlike radiofrequency ablation, it is not necessary to use a ground electrode for the more selective treatment of the lesion [16, 17]. The treatment of breast lesions is partly based on the dielectric properties of cancer tissue in comparison with healthy breast tissue. Cancer tissue contains a higher percentage of water content, favoring both electrical conductivity and permittivity of a magnetic field [18]. Previous research has demonstrated the possibility of applying this type of therapy to the treatment of noninfiltrating carcinoma, which manifests as a localized solid structure. The therapy involves the use of a coaxial slot antenna that functions as a waveguide for microwaves [19].

The article "Computational FEM Model and Phantom Validation of Microwave Ablation for Segmental Microcalcifications in Breasts Using a Coaxial Double-Slot Antenna" was published in 2021. Journal: Biomed Res Int.

Analysis of different factors, such as the frequency-dependent reflection coefficient (also termed the *S*_11_ parameter), is necessary to measure the efficiency of the used microwave applicator [20]. This coefficient reveals the amount of energy that is reflected from the antenna to calculate the standing wave ratio (SWR) factor, with which we can determine the mismatch of the antenna.

(1) $$\begin{array}{c} \;S_{11}=20\log10\left(\left|\Gamma \right|\right)=10\log_{10}\left(\frac{P_{\text{r}}}{P_{\text{in}}}\right)\left(\text{ⅆB}\right). \end{array}$$

Equation (1) represents the frequency-dependent reflection coefficient, where *P*_in_ is the input power and *P*_r_ is the power reflection (both given in W) [13]. This allows us to calculate the SWR by means of Equation (2), where Γ is the complex frequency-dependent reflection coefficient.

(2) $$\begin{array}{c} \text{SWR}=\frac{1+\left|\Gamma \right|}{1-\left|\Gamma \right|}. \end{array}$$

To calculate the reflected power in percent, the following formula is used:

(3) $$\begin{array}{c} P_{\text{r}}=100\;{\left|\Gamma \right|}^{2}\;\left(\%\right). \end{array}$$

Additionally, the specific absorption rate [3] defines the power absorbed by the tissues. This factor is useful in analyzing the radiation of nonionizing frequencies as shown below:

(4) $$\begin{array}{c} \text{SAR}=\frac{\sigma }{2\rho }{\left|E\right|}^{2}\left(\text{W}/\text{kg}\right). \end{array}$$

In this equation, *σ* is the tissue conductivity, *ρ* is the tissue density, and *E* is the electric field strength. The SAR parameter describes the increase in tissue temperature. The Pennes bioheat equation, given in Equation (5), defines the temperature distribution inside various tissues, considering the physiological factors that affect energy transfer. It is used to analyze the effects of electromagnetic waves on biological tissue.

(5) $$\begin{array}{c} \frac{\rho C\partial T}{\partial t}=\nabla \cdot \left(k\nabla T\right)\rho_{\text{bl}}C_{\text{bl}}\omega_{\text{bl}}\left(T_{\text{bl}}-T\right)+Q_{\text{met}}+Q_{\mathrm{ext}}. \end{array}$$

The Pennes bioheat equation is based on the thermodynamic characteristics of the blood to calculate heat accumulation in perfused tissue. In this equation, *ρ* is the tissue density, *C*_bl_ is the blood-specific heat capacity, *ω*_bl_ is the blood perfusion, *k* is the tissue thermal conductivity, *ρ*_bl_ is the blood density, C is the tissue-specific heat capacity, *T*_bl_ is the blood temperature, *T* is the final temperature, and *Q*_ext_ = *ρ*SAR (W/m^3^) is the external heat produced by the microwave antenna. Of note, *Q*_met_ is excluded because it is related to thermal variation due to metabolic activity, which is minimal during microwave ablation.

The article "Computational FEM Model and Phantom Validation of Microwave Ablation for Segmental Microcalcifications in Breasts Using a Coaxial Double-Slot Antenna" was published in 2021. Journal: Biomed Res Int.

Previous research demonstrated the possibility of performing microwave ablation therapy for breast carcinoma tissue [3]. Given the nature of the procedure (i.e., minimally invasive and replicable), it is important to explore possible applications for different types of lesions, such as premalignant lesions. Among these, microcalcifications stand out due to the threat they represent.

Breast calcifications are frequently observed through screening mammography in asymptomatic women. Most cases arise from benign processes, such as calcification of vascular structures, hyalinized fibroadenomas, cysts with apocrine changes, and ductal hyperplasia with or without atypia [21].

Calcifications of malignant origin result from central necrosis or secretions of malignant cells. They usually represent the only radiological sign of malignancy in asymptomatic patients, especially in those with calcifications that are not associated with the presence of a mass. Specifically, they are the only finding in most cases of ductal carcinoma *in situ* and in a smaller proportion of infiltrating carcinoma cases [22].

Mammography is the only imaging method capable of detecting malignant calcifications, far exceeding the ability of other methods for its detection in early breast cancer stages [23].

The Breast Imaging Reporting and Database System classifies calcifications according to their morphology and distribution. Regarding morphology, calcifications are categorized as typically benign, probably benign, and of suspicious morphology. With regard to distribution, calcifications are classified as diffuse, regional, grouped, linear, and segmental [24].

The aim of this study was to develop and compare a predictive computational model with a breast phantom, which emulates the dielectric properties of breast tissue with segmental microcalcifications. The frequency-dependent reflection coefficient and SWR factor were obtained to study the application of electromagnetic ablation to premalignant lesions in the breast, specifically segmental microcalcifications.

The article "Computational FEM Model and Phantom Validation of Microwave Ablation for Segmental Microcalcifications in Breasts Using a Coaxial Double-Slot Antenna" was published in 2021. Journal: Biomed Res Int.

A phantom is an object typically used for the calibration of MRI equipment. Different substances are used during the manufacture of phantoms to emulate specific characteristics of human tissues. In the case of the breast phantom used in this study, the intention was to emulate the dielectric properties of the tissue (i.e., conductivity and permittivity) rather than the physical properties related to obtaining diagnostic images.

The materials used to produce this phantom were tridestiled water, agarose, corn oil, neutral detergent, and tricalcium phosphate Ca_3_(PO_4_)_2_. Tridestiled water does not contain minerals or residual material; thus, it was used as a solvent. Agarose was used as a binder for the substances that comprise the phantom. Corn oil was used to emulate the properties of breast adipose tissue. The neutral detergent was added to homogenize all the elements of the mixture. Tricalcium phosphate is present in breast microcalcifications [25]; hence, it was used to perform the impurification of the phantom of breast tissue. It is agglutinated with water to generate small punctate clusters (see Figure 1) that are later randomly distributed throughout the whole phantom of breast tissue. Through this approach, we can emulate the distribution of microcalcifications in the breast (see Figure 2).

The phantom was produced according to the proportions shown in Table 1.

Measurements of the dielectric properties of isolated calcium phosphate (with a dielectric probe kit model 85070E) and SWR factor of the microcalcification phantom (with an open-ended coaxial probe model kit 5989-0222EN) were performed on an E5071B network analyzer ENA (Agilent, Colorado, USA). Measurements were taken at three different points with this probe using a support designed to keep the tip 70 mm away from the bottom of a 400 ml beaker (height: 107 mm)—this was the point where the highest concentration of tricalcium phosphate was found (see Figure 3).

Subsequently, in the same positioning, measurement of the SWR factor was performed using a coaxial double-slot antenna (see Figure 4).

It was decided to use a coaxial double-slot cable antenna because the radiation lobe is ideal for the ablation zone to cover the cluster of segmental microcalcifications due to the distribution in which they occur; besides, it has shown better results in previous studies [14], and it is easy to construct.

The antenna was wrapped with polytetrafluoroethylene tape to emulate the catheter, which would be introduced with a puncture to the breast during ablation therapy of biological tissue.

The microwave antenna used to perform the tests consisted of a microcoaxial cable with a diameter of 2,197 mm, which has an external copper conductor and an internal conductor of silver-plated copper separated by a polytetrafluoroethylene dielectric as shown in Figure 5.

The article "Computational FEM Model and Phantom Validation of Microwave Ablation for Segmental Microcalcifications in Breasts Using a Coaxial Double-Slot Antenna" was published in 2021. Journal: Biomed Res Int.

The antenna measurements according to the manufacturer and its dielectric properties are shown in Tables 2 and 3.

For both simulation and experimentation, the antenna operating frequency of 2.45 GHz was considered the frequency of interest. This frequency is part of the industrial, scientific, and medical band provided by the International Telecommunication Union, which is available worldwide for medical applications. Using this frequency, the effective wavelength in the tissue was calculated by means of the following equation [28]:

(6) $$\begin{array}{c} \lambda_{\text{eff}}=\frac{c}{f\sqrt{\varepsilon_{\text{r}}\mu_{\text{r}}}}. \end{array}$$

In this equation, *c* is the speed of light in free space, *f* is the frequency of the microwave generator feeding the needle applicator, *ε*_r_ represents the relative permittivity of the medium, and *μ*_r_ is the magnetic relative permeability of the medium. With these properties, the obtained wavelength values are shown in Table 4.

With these wavelength values, the maximum element size for the electromagnetic simulation can be obtained since it should be smaller than 1/8 of the effective wavelength; however, they should only be considered an approximation since the tissue properties are heterogeneous.

The simulation was performed using the COMSOL Multiphysics® 5.4 software [29] through the finite element method (FEM) to develop a three-dimensional model. This model consisted of a 70 mm radius sphere that represented the breast tissue, a double-slot antenna, and spiculated material that represented a premalignant lesion distributed as segmental microcalcifications (see Figure 6).

All empty space inside the sphere was considered breast tissue, while everything outside the sphere was considered air. The mesh of the geometry for the FEM analysis had a maximum element size of 24.47 mm, a minimum element size of 0.1191 mm, 470,396 vertices, 47,556 edges, 277,0381 elements, and a total volume computational domain equal to 1,392,000 mm^3^ (see Figure 7).

Table 5 shows the conditions under which simulation of the model was performed. The dielectric properties of the tissue and microcalcifications were maintained constant throughout the simulation.

## 3. Results

Figure 8 shows the temperature at the tip of the antenna for both computational models with and without blood perfusion; notice that the maximum temperature reached is higher in the model without perfusion.  Figure 9 presents the distribution of the heat generated in the heterogeneous tissue with an input power of 15 W after a treatment time of 500 s. The isothermal zone of 55°C is highlighted in green. This was the area in which breast tissue destruction was achieved because of the increase in temperature. The graph shows the complete 3D distribution in three axes. This process was repeated with and without blood perfusion to compare the findings with the results of the experimentation. Moreover, another computational model that considered these factors was subsequently produced.

The article "Computational FEM Model and Phantom Validation of Microwave Ablation for Segmental Microcalcifications in Breasts Using a Coaxial Double-Slot Antenna" was published in 2021. Journal: Biomed Res Int.

The blood perfusion rate, the specific heat of the blood, and the density of the blood were considered to analyze the difference in the temperature reached compared with the control simulation and the experiment using the tissue-mimicking phantom.

In the model, where blood perfusion is considered, the area of ablation was notably reduced. The maximum temperature between the two simulations achieved a level of 28.7°C. The SWR values obtained for the simulations and the experiment with the phantom are shown in Table 6.

Figure 10 shows a frequency sweep of 1–3 GHz. This in order to analyze the antenna characteristic resonance which is found at a frequency of 2.36 GHz with a *P*_r_ of -13.46 dB.

Figure 11 shows the *S*_11_ parameter for the computational model and the validation experiments; the bandwidth was reduced to focus near the analyzed operation frequency. It is important to notice that the antenna coupling is better in the experiment than in the computational model.

## 4. Discussion

The SWR values in the three measurements exhibited a change of 0.191 between the minimum and maximum SWR and –1.76 in *S*_11_ obtained values, implying a variation of power reflection of 2.8%. Comparison of the average of the three measurements with the values of the simulations yielded a SWR difference of 0.064, representing a 0.9% difference in power reflection. The variation observed between the computational model and the experiment with the phantom is attributed to differences in the distribution of the microcalcifications.

This comparison allows us to determine the accuracy of the simulations performed using the COMSOL Multiphysics software. Blood perfusion is depreciated, as the phantom does not include this characteristic.

## 5. Conclusion

In conclusion, both experimentation using the phantom and simulations demonstrated that ablation therapy can be performed using this antenna; however, further investigation focusing on antenna optimization is warranted to reach the maximum possible efficiency and reduce the power reflection below the acceptable value of 1% before we can perform heating tests with biological tissue. It is also important to perform *ex vivo* test tests in various tissues to compare the temperature with the one obtained in the simulation since the phantom is not appropriate for this because of its melting point (approximately 50°C). The computational model shows good results despite the differences in the values; these variations are due to the difference in the microcalcification distribution and phantom anisotropy.

The article "Computational FEM Model and Phantom Validation of Microwave Ablation for Segmental Microcalcifications in Breasts Using a Coaxial Double-Slot Antenna" was published in 2021. Journal: Biomed Res Int.

## Figures and Tables

**Figure 1:** Tricalcium phosphate for mimicking microcalcifications.

**Figure 2:** Random distribution of microcalcifications in the breast tissue phantom.

**Figure 3:** Microcalcification phantom with three measuring points and dielectric coaxial open probe.

**Figure 4:** The coaxial double-slot antenna wrapped with polytetrafluoroethylene tape.

**Figure 5:** View of the axial cut of the double-slot antenna (measures are given in mm).

**Figure 6:** 3D geometric model of the antenna and breast tissue.

**Figure 7:** Mesh of the model of the antenna, breast, and microcalcifications.

**Figure 8:** Temperature at the tip of the antenna of both computational models with and without blood perfusion.

**Figure 9:** Comparison of temperature distributions of the breast model including microcalcification considering (b) and without considering (a) energy loss due to blood flow for different time moments (100 s, 200 s, 300 s, 400 s, and 500 s).

**Figure 10:** The *S*_11_ distributions (dB) for the computational model from 1 to 3 GHz.

**Figure 11:** The *S*_11_ distributions (dB) for the computational model and the validation experiment.

**Table 1:** Concentrations used for preparing the breast microcalcification phantom.

Materials	Concentration
Tridestilated water	50 ml
Agarose	4.5 g
Corn oil	160 ml
Neutral detergent	30 ml
Tricalcium phosphate	2.14 g

**Table 2:** Dimensions of the antenna elements [26].

Component	Diameter (mm)
External conductor	2.197 ± 0.0254
Dielectric	1.68 ± 0.0254
Internal conductor	0.51 ± 0.0127
Catheter	2.64 ± 0.03

**Table 3:** Dielectric properties of the antenna [14, 27].

Material	Relative permittivity (*ε*_r_)
Dielectric	2.03
Catheter	2.60

**Table 4:** Effective wavelength of phantom materials.

Material	*λ*_eff_ (mm)
Breast tissue	66.57
Tricalcium phosphate	60.99
Average	63.78

**Table 5:** Parameters used in the FEM simulation.

Parameter	Value	Reference
Input power, *P*_in_	12 W	—
Frequency, *f*	2.45 GHz	—
Electrical conductivity of breast tissue, *σ*_breast_	0.137 S·m^−1^	[29]
Thermal conductivity of breast tissue, *k*_breast_	0.42 W·m^−1^·K^−1^	[30]
Relative permittivity of breast tissue, *ε*_r,breast_	5.1467	[29]
Relative permeability of breast tissue, *μ*_r,breast_	1	—
Blood density, *ρ*_bl_	1040 kg·m^−3^	[30]
Specific heat of blood, *C*_bl_	3639 J·kg^−1^·K^−1^	[31]
Blood perfusion rate, *ω*_bl_	0.0036 s^−1^	[31]
Heat capacity of tricalcium phosphate at constant pressure, *C*_cf_	227.8 J·mol^−1^·K^−1^	[32]
Density of tricalcium phosphate, *ρ*_cf_	3140 kg·m^−3^	[33]
Thermal conductivity of tricalcium phosphate, *k*_cf_	0.612 W· m^−1^·K^−1^	[34]
Relative permittivity of tricalcium phosphate, *ε*_r,cf_	4.0296	Measured
Electrical conductivity of tricalcium phosphate, *σ*_cf_	0.1394 S·m^−1^	Measured
Relative permeability of tricalcium phosphate, *μ*_r,cf_	1	—

The article "Computational FEM Model and Phantom Validation of Microwave Ablation for Segmental Microcalcifications in Breasts Using a Coaxial Double-Slot Antenna" was published in 2021. Journal: Biomed Res Int.

**Table 6:** Comparison of *S*_11_, SWR, and *P*_r_ in analyzed models.

	*S*_11_ (dB)	SWR	*P*_r_ (%)
Measurement 1	–12.64	1.609	5.4
Measurement 2	–10.88	1.800	8.2
Measurement 3	–11.68	1.705	6.8
Simulated without blood	–12.30	1.641	5.9
Simulated with blood	–12.30	1.641	5.9
Measurement average	–11.68	1.705	6.8

Abbreviations: *S*_11_: reflection coefficient; SWR: standing wave ratio; *P*_r_: reflected power.

## Data Availability

The data used to support the findings of this study are included within the article.
